RETRACTED

# Application of Big Data Technology to Promote Agricultural Structure Adjustment and High-Quality Development of Modern Agriculture

**DOI:** 10.1155/2022/5222760

**Published:** 2022-09-29

**Authors:** Xiaoxian Ju

**Affiliations:** Henan University of Animal Husbandry and Economy, Zhengzhou 450046, China

## Abstract

The implementation of the strategy of rural revitalization is a major ministerial work made by the Nineteenth National Congress of the Communist Party of China and is the general grasp of contemporary agriculture, peasants, and rural work. In recent years, with the rapid development of remote sensing technology and deep learning technology, the demand for the technology for the classification of crops on satellite remote sensing images based on deep learning technology has increased in agricultural insurance and land survey. Therefore, this paper trains one, which is 85.9%–92.8%, the accuracy of corn classification is 77%–93%, and the accuracy of forest classification is 77%–87.6%. Subsequently, the overall accuracy of classifying all directories through the multi-temporal validation data set between May 2017 and October 2017 reached 92.6%. Such a multi-time combination method can be used for monthly, timely, and efficient iteration of agricultural insurance and crop yield estimation, which will be more accurate each time. These methods can also be further applied to the growth and change monitoring of large agricultural planting areas, adding bricks and tiles to China's agricultural remote sensing. If the countryside is to be revitalized, agriculture must develop rapidly at the same time, industries must flourish, ecology must be livable, rural customs must be civilized, and life must be prosperous. Modern agriculture is a comprehensive circulation system with high yield, high quality, low consumption, ecology, environmental protection, and high efficiency. The development of modern agriculture is inseparable from the industrialization of agriculture, the globalization of agriculture, the digitization of agriculture, the integration of agriculture, the adjustment of agricultural structure, and agricultural innovation. Only the continuous development of modern agriculture can make rural revitalization enter a new journey.

## 1. Introduction

China is now a powerful agricultural country with 1.4 billion people. Agricultural products determine the social value of grain and directly affect the living level of people [1]. Grain production is related to national transportation and people's livelihood, which is the basic consensus of this paper. Food production needs to ensure safety [2] All these are important sources of our sense of security. The mountains are green, the forest is stone, and the world is safe. Since 2004, China's grain production has continued for 16 years, with a bumper harvest every year [3]. At present, the state vigorously promotes the strategy of rural revitalization, and leading cadres at all levels are actively committed to optimizing rural formats, especially taking the reorganization of various resources as the starting point, actively using the advantages of land, space, labor, and other advantages to vigorously develop modern agriculture and help rural revitalization.

RETRACTED

The latest opinions on food security issues were put forward at the second National Congress in 2020 [4]. According to the principle of “ensuring the basic self-sufficiency of grain and the absolute safety of rations,” the government has formulated the agricultural policy of putting people first, maintaining the balance of domestic and foreign demand, insisting on expanding production, appropriately liberalizing the customs of some agricultural products, and importing domestic crops of grain [5]. Scientific and technological development is an important strategy for China's food security. We will always adhere to the path of food security with Chinese characteristics. Under the epidemic situation in 2020, the country and society mentioned in the text will still maintain stable social order, but the safe supply of agricultural products and food will still be improved [6]. Under the premise of changes in the external environment, the country's economic development will remain relatively stable. Through their own agricultural development, the Chinese people have not only maintained the stability of the people's production but also maintained the foundation for national economic recovery. Therefore, the stablility of agricultural structure and the high-quality development of the modern agricultural system are indispensable [7].

Annual crop conditions play a significant role in harvest. Determining the maturity of grain crop coverage plays an important role in promoting national food security and the sustainable development of the rural economy. Through macro-control, China can understand the situation of crops and select various types of cultivation methods. Adapt to the growing needs of mankind and the ever-changing production requirements [8]. The countryside must be revitalized, not without agriculture. To develop agriculture, is impossible to do without the progress of agricultural science and technology, without the training of professional farmers, and even more without the innovation of agricultural production and management.

In the practice of agricultural land use, the situation of crop planting land in China is very complicated. The landforms such as flat land, mountains, and hills are variable and undulating with a large span. In the plain area, some land is suitable for large-scale or intensive agricultural production; in the hilly area, it is suitable for fruit cultivation or returning farmland to forest; in the mountainous area, it is suitable for developing green planting. However, only by rationally developing the planting industry according to different terrain can we promote the healthy and sustainable development of rural areas [9]. Under the interference of various reasons, China's agriculture is facing great historical challenges. Under this premise, only by finding the right way can China's agricultural products greatly improve their output efficiency [10].

RETRACTED

If statistical analysis is carried out only by the manual measurement method, its cost is quite expensive and cannot be popularized, because it requires a large number of locally collected survey data and a large number of manual operations. Land statistics based on big data analysis is a modern scientific research method [11]. For example, the complex model represented by in-depth learning can automatically obtain agricultural environmental information and automatically adjust the industrial structure through learning a large number of remote sensing satellite image data, which can not only save labor costs and time costs but also maximize benefits [12]. Therefore, agriculture should focus on diversified development, and high-quality links should be carried out with new village planning, new industrial development, cultural reinheritance, etc., so that modern agriculture can show a thriving development outlook. China is a large country with a vast source and very rich agricultural resources and a large agricultural population is large, so to rejuvenate the Chinese nation, we cannot but attach importance to agriculture, and only with the modernization and development of agriculture can we have the smooth realization of rural revitalization.

## 2. State of the Art

### 2.1. Modern Agricultural Digitalization

Modern agricultural digitalization includes high-tech electronic intelligent control equipment such as seedling breeding, cultivation management, soil, and environmental management, so that agricultural production methods can achieve intelligent management, remote diagnosis, remote control, and disaster early warning.

The application of deep learning technology in agricultural remote sensing analysis is , and crop classification methods will be increasingly diverse. Historically, different forms of deep learning have had a great impact on crop coverage surveys. More satellite data are now easier to obtain than in the past [13]. The use and construction of large digital changes for the countryside. Zero people think that deep learning technology is very important for remote sensing data processing, especially in the era of remote sensing big data processing [14]. Deep learning technology will become the most advanced biological remote sensing technology. With the help of remote sensing big data analysis, *s* zero can provide services for fine agriculture through deep cognition technology. Specifically, by applying the semantic segmentation mode, crop information can be obtained more efficiently in remote sensing video. Based on the difference of crop species, the semantic segmentation mode can also get the marks of each pixel in the remote sensing image. Remote sensing semantic division is often used in agricultural image classification [15].

RETRACTED

Based on the richness of remote sensing data, the main task is to identify nonRGB images because such images not only contain RGB bands but also other bands in the image data. It is extremely difficult and flexible to make all the effective bands in remote sensing images [16]. Li. Extracted rice fields using a multi band medium high resolution image spectrometer (MODIS). In addition, Huang. Also used the ones. These two studies use more RGB signals than traditional remote sensing image processing. With the continuous movement of the moon in the sky, it can continuously obtain a large number of multi-temporal images. In this paper, multi-temporal data can also be used to observe the change of landforms or crop growth [17]. For example, it can monitor the ecological diversity of grassland vegetation and even eliminate the impact of clouds in remote sensing images. All these functions can be realized with the help of more time phase diagrams. This facilitates the practical application of multispectral remote sensing images in this paper [18].

At present, China's agriculture has entered a new stage of high-quality development, in accordance with the new requirements of high-quality development, it is necessary to accelerate the pace of modern industrialized agricultural development and further promote the integrated development of primary, secondary, and tertiary industries. First, it is necessary to expand in terms of resources, markets, business formats, and products; second, it is necessary to do a good job in combining agriculture and leisure tourism, agriculture and circulation culture, agriculture and healthy old-age care, and agriculture and local education; the third is to realize the integration of various business forms and the complementary advantages of various business forms.

RETRACTED

However, there are still a number of problems that must be overcome. Therefore, if people want to use the full band signals and multi-phase signals of satellite images at the same time, it is necessary to investigate how computers can carry such large-scale data processing in the process of deep learning training. Although single-phase remote sensing images are easy to obtain, the image sequences for geographical coordinates. An effective multi-temporal semantic segmentation model requires a large amount of temporal information training. So, of course, another way to add training data is also. Therefore, we must find a way to study how to train a good multi-time-related semantic segmentation mode without abundant temporal information [19].

### 2.2. Multi Temporal Remote Sensing Satellite Image

With the development of remote sensing technology, the spatial clarity of satellite remote sensing images has been gradually improved, so that people can more accurately obtain the actual data in remote sensing images. World rural development is the basic outlet and inevitable development of rural areas. Its basic purpose is to make full use of the advantages of all kinds of modern agricultural products in the world, deeply participate in global rural cooperation, optimize the allocation of agricultural product resources, expand the supply of modern agricultural products, and further improve the income of farmers.

At present, there are mainly three kinds of analysis technologies used in multispectral remote sensing, namely, semisupervised classification technology, supervised analysis technology and nonsupervised analysis technology. Semisupervised classification technology mainly includes selftraining, joint training, semisupervised vector method and traditional naive Bayesian classification. 2. Unsupervised methods are mainly divided into some clustering methods and principal component methods, such as k-means clustering method and the PCA linear dimension reduction method. The supervised method is the most common classification method, and the neural network method is the most common. In addition, there are the Mahalanobis distance judgment method, Fisher: linear judgment method, second normal form distance judgment method, and so on [20].

### 2.3. Semantic Segmentation Neural Network

The convolution layer: since people can obtain information about images by convolution operation, the.

Some features of the original signal are enhanced, and noise is reduced. As shown in Figure 1, by mapping the input to the input, taking filter: as the convolution kernel and (1) as the convolution operation, we can obtain the results of all the feature maps in the figure. The results of feature mapping can be used as feature maps in neural networks.

(1) $$\begin{array}{c} \left(f*g\right)\left(n\right)=\sum_{0}^{\infty }\left(f\left(x\right)*g\left(n-x\right)\right)\text{.} \end{array}$$

Full connection layer: many-to-many mapping is adopted for each input and output, and multi-dimensional signals are mapped to the entire output layer through SoftMax parameters. SoftMax can be used to obtain the corresponding confidence of all input and output data in this article. The standard expression of the SoftMax parameter is equation (2). Where *X* represents the output framework of the upper layer of the model, *Y* represents the final division conclusion of SoftMax, and *wi* is the weight value of this layer.

(2) $$\begin{array}{c} p\left(y\;|\;x\right)=\frac{\exp\;\left(W_{y}\cdot x\right)}{\sum_{C=1}^{C}\exp\;\left(W_{c}\cdot x\right)}\text{.} \end{array}$$

RETRACTED

### 2.4. Loss Function

The loss function is used to measure the difference between the simulated predicted value and the actual label value (ideal output value). Generally speaking, the loss function directly affects the quality of simulation. The loss function generally includes two compopnents: experience risk loss function and structural risk loss function. The structural risk loss function refers to the empirical risk loss function plus the regular term. Realize the further exchange of agricultural products and labor to form an interconnected global whole; the second is to actively do a good job in international agricultural technology exchanges and cooperation, and take the initiative to exchange and dock global high-tech achievements; the third is to reform the traditional farming mode and develop organic agriculture and ecological agriculture; the fourth is to increase cooperation in the global market to realize the operation of agricultural commodities in the world.

Common loss functions are 0-1 loss functions, that is, the correct value is 1 and the error value is 0. The 0-1 loss function is usually used to judge the number of errors and is not suitable for fitting the real difference results. As formula :

(3) $$\begin{array}{c} L\left(Y,f\left(X\right)\right)=\left\{\begin{array}{c} 1,Y\neq f\left(X\right)\\ 0,Y=f\left(X\right) \end{array}\right.\text{.} \end{array}$$

The absolute value loss function can describe the deviation of the calculation results in the one-dimensional straight line, as shown in formula :

(4) $$\begin{array}{c} L\left(Y,f\left(x\right)\right)=\left|Y-f\left(x\right)\right|\text{.} \end{array}$$

Log loss function is also one of the most commonly used loss functions. This logarithmic function can also well describe the difference between numerical distribution results. It is a loss function used when analyzing scenarios and is used to describe various types of confidence quantities. However, it has high robustness but poor robustness to noise. and the robustness against noise is poor. Formula (2) five

(5) $$\begin{array}{c} L\left(Y,P\left(Y\;|\;X\right)\right)=-\log\;P\left(Y\;|\;X\right)\text{.} \end{array}$$

The square loss function is often used in regression and pixel-level prediction. It is easy to calculate, but the weight update is slow. It can better express the direct difference between the output value and the predicted value:

(6) $$\begin{array}{c} L\left(Y\;|\;f\left(X\right)\right)=\exp\;\left[-yf\left(x\right)\right]\text{.} \end{array}$$

Cross entropy loss function, such as 2 7. It is mathematically known as the likelihood function. When the calculation of the square difference function is slow, this paper usually uses the cross line to calculate the function. It is often used in multi-classification tasks. In this paper, softmax is used as the activation parameter of the output method, and the cross entropy loss method is generally used. It can overcome the phenomenon that the weight adjustment speed of the square loss function is slow, and it can also automatically adapt to the update according to the error degree:

(7) $$\begin{array}{c} C=-\frac{1}{n}\sum_{x}\left[y\;\ln\;a+\left(1-y\right)\ln\;\left(1-a\right)\right]\text{.} \end{array}$$

RETRACTED

### 2.5. U-NET

The U-net network is a classical semantic segmentation neural network, and its two sides are symmetrical. It is a standard neural network with an encoder decoder architecture. It can complete end-to-end image mapping, such as the basic structure of u-net shown in Figure 2. As an extension of the FCN network, the u-net network can also be applied to the case where the amount of marked data is relatively small. In general, the number of labeled data for medical data is relatively small, so u-net can better meet the training of small sample number. The u-net network integrates the feature structure information in the down sampling process into the up sampling process through the integration method, so that the coordinate signals in the original image features can be more accurately retained.

## 3. Methodology

The Deeplab network is a series of network structures proposed by Hekaiming and others. It is also a common and practical network structure in recent years. From the deeplab V1 network to today's deeplab v3+ network, the accuracy of the deeplab network in semantic segmentation has been greatly improved.

The overall structure of the deeplabv3+ network is shown in Figure 3 It is also a network model of the encoder-decoder structure. The encoder part of the network uses the entire deeplabv3 network model and the DCNN (deep convolutional neural network) Generally, only the convolutional neural network of the RESNET system can be used. The architecture adopts the ASPP architecture and introduces multi-scale image signals. In the decoder part, the deep labv3 + network combines the low-level characteristic signal of the deep labv3 network with the high-level characteristic signal output by the deep labv2. Then, the conclusion is obtained by convolution calculation. To promote a new round of high-quality industrial revitalization in Dongtai rural areas, it is necessary to further emancipate the mind, based on the further implementation of the national agricultural modernization revitalization policy and the demand for agricultural and rural high-quality industries, and adhering to the government's purpose of serving agriculture and the people's livelihood, conscientiously shoulder the responsibility of industrial revitalization, actively seek new problems, pay close attention to policy implementation, implement the concept of integrated development of three industries and the idea of full value chain development. Great progress has been made in the fields of quality brand building and green industry development. We will actively integrate the primary, secondary, and tertiary industries in rural areas, reform and open up new development, and vigorously promote agriculture and rural high-quality industries.

RETRACTED

A satellite image is a very convenient tool for agricultural investigation. With the progress of deep learning, this paper can use the method of deep learning to learn crops. In the business of agricultural insurance, in-depth learning technology and skills are used to effectively extract the planting areas and types of crops, which can quickly produce results and save human costs. Policy innovation is the power source of rural industrial revitalization, and policy guarantee is the driving force of rural industrial revitalization. First, comprehensively promote agricultural reform. We should grasp the relationship between top-level design and basic exploration, overall integration and key breakthroughs, solidly promote the reform of the rural “Three Rights Separation,” the collective property rights system and the rural financial system, accelerate the structural transformation of the rural supply side, and further improve the input system for agricultural economic development.

The main data collection area of this paper is Jilin, which is located in the center of Northeast China, adjacent to Daliao Province, Inner Mongolia, Heilongjiang Province, the Russian Federation and South Korea. It is also the main geographical center of Northeast China studied in this paper, and the regional shape changes significantly. From the perspective of landform, the landform is inclined from southeast to northwest of Jiangsu, showing the characteristics of high in the southeast and east and low in the northwest of Jiangsu. The whole province can be divided into two types of terrain: the eastern hills and the central and western alluvial plains. Jilin is the main grain and oil production province in China. By 2019, the sown area of grain and oil will be 5.645 million hectares, including 840 hectares of rice, 400 hectares of wheat, 421.5 hectares of corn, and 1 million hectares of wheat 1996. The cumulative total output of grain and oil was 38.78 million tons.

RETRACTED

In such an important area, in order to ensure that the growth of crops can be monitored and farmers can plant crops at ease, the state has implemented an agricultural insurance policy for major crops. The main purpose of this paper is to monitor and extract these planting areas.

The data in this paper is from the remote sensing satellite Landsat 8, launched by the United States in 2013. It is equipped with an oli land imager to detect the soil, and a TIRS thermal infrared sensor to detect the infrared spectrum information of the sun. This paper mainly uses its old method. Oli is divided into nine beams, as shown in Table 1.

## 4. Result Analysis and Discussion

The neural network architecture used in this experiment is very complex, and it must rely on more powerful technical computing power than the GPU. In this paper, the PyTorch framework based on CUDA will be used to recode the program. The machine configuration used in this article is shown in Table 2:

This paper uses the oli part of landsat8, which is a part of multispectral data and consists of 7 channels.

We can train the data set in this paper through deeplav3 +, deeplav3 and the u-net network. In the preset weight part of the training system, we can initialize the DCNN part of the system with the magenet pretraining weight. One of the learning rates is the default starting point of the system, which is 50 rounds, that is, the learning rate is 0 1, 0 01, 0 001, 0 0001 in descending order. The optimizers of the three networks are designed as SGD (gradient descent algorithms), and the loss function uses the cross-entropy loss function. According to the new needs of economic construction, we will intensify the development of modern agricultural products and continue to promote the integration of primary, secondary, and tertiary industries.

### 4.1. Evaluation of Experimental Results for Three Different Models

This paper can clearly observe that the convergence speed and accuracy of the deeplabv3+ network are higher than those of the other two networks. Compared with the original deeplabv3 network, the deeplabv3+ network can more effectively combine the low-level features and high-level features. In Figures 4 and 5 It can be seen from Figure 4 that the deep lavv3+ network has obvious convergence speed and accuracy.

RETRACTED

Higher than the other two networks.

In this paper, the data set from May to the end of September 2017 is divided into four stages according to the growth and development stages, mainly because the crop characteristics of the four stages are quite different. There is a very simple neural network modeling for each data set. The DCNN module of Deep Labv3 + is used to replace the network model in this paper. First, taking the above SE model as an example, the attention model is directly referred to the network structure of ResNet. This chapter uses ResNet to compare with the three-depth ResNet system. The experimental results are shown in the following Table 3:

In the above table, it is obvious that the performance of Se ResNet network is slightly higher than that of other networks.

### 4.2. Crop Classification Using Multi Temporal Remote Sensing Data Based on Posterior Probability

The model trained based on a single time period is limited in its actual process. We always look forward to finding a way to break from the traditional method of determining crop types based on one month's survey. Our hope is that we can judge the types of crops within a specific range through several months of investigation and research, or prepare remote sensing maps of a region through many remote sensing satellites many times, so as to make the conclusion more credible.

The training idea of multi temporal image data is usually to align the remote sensing images taken by satellites at different time points for a single geographical coordinate region. That is to say, the training images must be in the same time dimension, and ensure that the same crops are logically consistent in the image pixel coordinates under the same geographical coordinates. Logically, such clipping is described to assume that there are clouds in the picture. Therefore, according to the logic of the neural network, the clipping here belongs to an unknown type, which will lead to mismatching with the image coordinates of the target position. Of course, a few errors can be tolerated, but a large number of errors always occur in actual operation.

### 4.3. Single Phase Division of Multi-Phase Data

Due to the limitation of Superposition Technology in integrated training, and considering the difficulty of training large time phase data sets, this chapter presents a single time training method and a step-by-step method of final synthesis. According to the growth process of these crops, the training of large temporal data sets includes four disjoint stages. In this way, we can use these data separately in the way in Chapter 3. Then, this paper trains these models with four sub-methods and summarizes the results of simulation training with some of these methods.

RETRACTED

The first is the division of data sets. In this paper, the data set is divided according to four growth time stages, and the results in the following table are obtained. Each image is divided into 512 × 512 × 7 sizes. Then, the four basic models are trained according to the data in the following table. Similar to the third chapter, the paper adopts three semantic segmentation modes, namely u-net, deeplav3, and deeplav3 + network. The posterior probability of each model prediction, the article also saves as 20% of the experimental data as the test set, and the test set does not participate in the model exercise.  Table 4 shows the total amount of data collected for training.

After basic data separation, this paper can get four groups of separated models. How to merge the models according to stacking's integrated learning method in the prediction stage?

It notes the corresponding simple equilibrium and weighted average, meta learning method. Although the above method is simpler and more convenient than the method based on its average value, the overall effect will be low. Because it is easy to receive the effect of the shortcomings of a single model by using this model, the models have their own advantages in compounding. This chapter gives a model compounding method based on a posteriori probability:

(8) $$\begin{array}{c} H\left(x\right)=\underset{j}{Argmax}\overset{i=1}{\underset{4}{\sum }}g\left(y_{j},h_{i}\left(x\right)\right)\text{,}\\ g\left(y_{j},h_{i}\left(x\right)\right)=P\left(y_{j}\;|\;h_{i}\left(x\right)\right)\text{,}\\ y=f\left(W\cdot d\left(x\right)\right)\text{.} \end{array}$$

The each mode operation, indicates the conditional, that is, when the predicted value is *h* (*x*), the actual real number is *Y*_*J*_. By adding the accumulated pixel values of the target area through multiple modules according to the weight, the predicted value of the target area can be obtained.

In this paper, the four models are trained in data sets, and it is found that the deeplabv3+ network.

Maintain the best performance in the. Based on the deeplabv3+ model, this paper tests the accuracy of the test set, as shown in Table 5.

This table is its corresponding test set to indicate the posttest probability value of each model under its own classification. From the perspective of posttest probability, the method in this paper will help to highlight the highest probability results in the classification results. Therefore, it can be assumed that the classification result of a model is rice, but it may also be wheat or forest land, although the probability is not very high. However, this paper has obtained the accuracy of the prediction results of various crops in each model from the actual test set and used it as the posttest probability. Among the classification results of the specified patterns, the posttest probability results are also very effective.

RETRACTED

## 5. Conclusion

In order to overcome the limitation of the single period model in the practical production process, this paper also proposes a multi-temporal remote sensing data division based on a posteriori probability. The development of agricultural modernization and the implementation of the strategy of comprehensive rural revitalization have enabled modern agriculture and rural revitalization to enter a new stage of development in an all-round way. Only when we firmly follow the road of development with Chinese characteristics in the new era, proceed from practical problems, follow the path of socialist construction of new rural areas, new agriculture, and new rural areas, and realize the transformation and upgrading of modern agriculture from traditional Chinese rural areas, can we certainly achieve the modernization of Chinese rural areas, and achieve comprehensive rural revitalization.

In addition, because the probability analysis is discrete, the information in the control process is iterated once a year. In this way, as the crop growth cycle continues to change, the model will help to integrate the information of each growth cycle in the growth cycle. In addition, the Superposition Technology of the model can also tolerate the information loss in a specific period, such as the above effects brought by cloud coverage and long satellite return periods.

## Figures and Tables

**Figure 1:** Principle of convolution operation.

**Figure 2:** The basic structure of a U-net network.

**Figure 3:** Structure diagram of the DeepLabV3+ network.

**Figure 4:** Loss graph.

**Figure 5:** Accuracy graph.

**Table 1:** Introduction to oli parameters of Landsat 8 satellite.

Band	Pixel resolution (m)	Wavelength range (*μ*m)	Main applications
Band 1 coastal	30	0.433–0.453	Shoreline observation
Band 2 blue	30	0.450–0.515	Water penetration
Band 3 green	30	0.525–0.600	Basic discrimination of vegetation
Band 4 red	30	0.630–0.680	Chlorophyll absorption degree
Band 5 NIR	30	0.845–0.885	Distinguish the wetness of the land
Band 6 SWIR 1	30	1.560–1.660	Distinguish bare ground
Band 7 SWIR 2	30	2.100-2.300	Discrimination of rocks and minerals
Band 8 pan	15	0.500–0.680	Enhanced resolution
Band 9 cirrus	30	1.360–1.390	Cloud detection usage

RETRACTED

**Table 2:** Equipment configuration.

Project	Content
Central processing unit	Intel(R) core(TM) i7-7700K CPU @ 4.20 GHz
Memory	128 G
Graphics card	2 ^*∗*^NVIDIA GeForce GTX 1080Ti
Operating system	Ubuntu16.04
CUDA	Cuda10.0 with cudnn
Data processing	Python3.7, pytorch

**Table 3:** Comparison of experimental data collected under different network structures in different stages.

Name	SE-ResNext101	ResNext101	ResNet50	ResNet101	ResNet152
Data part l	90	89.3	87.7	88	84
Data part 2	85.7	84.1	84.9	83.4	84.7
Data part 3	88.1	82.5	84.5	87.8	87.6
Data part 4	88.7	85.7	86.45	86.3	86.6

**Table 4:** Data volume in the data set of each time period.

Dateset sub-part	Amount
Part 1	848
Part 2	992
Part 3	1072
Part 4	1328

**Table 5:** Confusion matrix obtained on the test set by Deepl abv3+ model of each training set.

	Ture	Prediction			
	Label	Rice	Com	Forest	Other
Part 1	Rice	0.883	0.017	0.038	0.062
	Corm	0.096	0.776	0.093	0.034
	Forest	0.098	0.027	0.777	0.097
	Other	0.043	0.004	0.033	0.92

Part 2	Rice	0.928	0.037	0.024	0.011
	Corn	0.076	0.803	0.069	0.052
	Forest	0.117	0.123	0.741	0.019
	Other	0.015	0.013	0.007	0.964

Part 3	Rice	0.859	0.007	0.103	0.03
	Corn	0.117	0.771	0.1	0.011
	Forest	0.217	0.026	0.744	0.011
	Other	0.047	0.002	0.007	0.945

Part 4	Rice	0.86	0.042	0.083	0.015
	Corn	0.062	0.934	0.003	0.001
	Forest	0.116	0.001	0.876	0.006
	Other	0.121	0.009	0.033	0.836

## Data Availability

The labeled dataset used to support the findings of this study are available from the corresponding author upon request.

## References

[1] Desconsi C. (2020). The production of development expectations and the pace of agricultural expansion: analysis of land-use practices by small farmers in northern Mato Grosso State – Brazil. *Caderno de Geografia*.

[2] Gomez A., Narayan M., Zhao L. (2020). Effects of nano-enabled agricultural strategies on food quality: current knowledge and future research needs. *Journal of Hazardous Materials*.

[3] Nye C. (2020). Agriculture’s “other” contingent labour source. Agricultural contractors and relationships of interdependence at the farmer-contractor interface. *Journal of Rural Studies*.

[4] Kamari S., Ghorbani F. (2021). Extraction of highly pure silica from rice husk as an agricultural by-product and its application in the production of magnetic mesoporous silica MCM–41. *Biomass Conversion and Biorefinery*.

[5] Grigorescu I., Dumitric C., Dumitracu M. (2021). Urban development and the (Re)use of the communist-built industrial and agricultural sites after 1990 the showcase of bucharest–ilfov development region. *Land*.

RETRACTED

[6] Oblova I., Gerasimova I., Sishchuk J. (2020). Case-study based development of professional communicative competence of agricultural and environmental engineering students. *E3S Web of Conferences*.

[7] Teplova L., Chuikova V., Afanasyeva L. (2020). Agricultural consumer credit co-operations one of the most important resources for the development of small and medium business. *Russian Journal of Management*.

[8] George T. (2020). A new look at agricultural development and the non-agriculture economy in low-income countries. *Global Food Security*.

[9] Mazur K. (2020). Innovative development of the agricultural market: research of modern tendencies and strategies. *Eсonomy finanсes management Topical issues of science and practical activity*.

[10] Subota M., Demydova M. (2020). Modeling of processes of providing high-quality sanatorium and resort services as a precondition for sustainable development of enterprises. *University Economic Bulletin*.

[11] Zhukova T., Panfilova O., Avlasenko I., Avlasenko L. (2020). Peculiarities and development factors of modern agricultural engineering. *E3S Web of Conferences*.

[12] Medvedeva L. S. (2020). The development of agricultural export through the generation of high quality analytics. *IOP Conference Series: Earth and Environmental Science*.

[13] Gu H. y., Wang C. w. (2020). Impacts of the COVID-19 pandemic on vegetable production and countermeasures from an agricultural insurance perspective. *Journal of Integrative Agriculture*.

[14] Payero J. O., Marshall M. W., Nafchi A. M. (2021). Development of an internet of things (IoT) system for measuring agricultural runoff quantity and quality. *Agricultural Sciences*.

[15] Demetrio P. M., Rimoldi F., Peluso M. L. (2022). Impact of intensive agricultural production on the ecotoxicologic quality of associated medium-order streams: cereal and oilseed versus horticultural production. *Environmental Management*.

[16] Chymosh K. (2020). Analysis of modern world and domestic trends in the development of transport logistics in the agricultural sector of the economy. *Ekonomika ta Derzhava*.

[17] Gervais A., Fournier V., Bélisle M. (2020). Agricultural landscape composition affects the development and life expectancy of colonies of Bombus impatiens. *Ecosphere*.

[18] Costa J. R., Tonon R. V., Cabral L. (2020). Valorization of agricultural lignocellulosic plant by-products through enzymatic and enzyme-assisted extraction of high-added value compounds: a review. *ACS Sustainable Chemistry & Engineering*.

RETRACTED

[19] Raza M., Lee J. Y. (2022). Relationship between agricultural land use and spatial heterogeneity in quality of water resources in haean basin of korea. *Water Resources*.

[20] Petrova O. G., Malkhasyan A. B. (2021). On the need for state support for the development of rural tourism as a type of non-agricultural activity in the Pskov Region. *IOP Conference Series: Earth and Environmental Science*.

